The article "Deep Scale-Variant Network for Femur Trochanteric Fracture Classification with HP Loss" was retracted in 2023. Reasons: signs of a paper mill; compromised peer review; unreliable results or conclusions.

# Deep Scale-Variant Network for Femur Trochanteric Fracture Classification with HP Loss

**DOI:** 10.1155/2022/1560438

**Published:** 2022-03-27

**Authors:** Yuxiang Kang, Zhipeng Ren, Yinguang Zhang, Aiming Zhang, Weizhe Xu, Guokai Zhang, Qiang Dong

**Affiliations:** ^1^Department of Orthopaedics, Tianjin Hospital, Tianjin 300211, China; ^2^School of Optical-Electrical and Computer Engineering, University of Shanghai for Science and Technology, Shanghai 200093, China; ^3^School of Computer Science, The University of Manchester, M14 5ta, Manchester, UK

## Abstract

Achieving automatic classification of femur trochanteric fracture from the edge computing device is of great importance and value for remote diagnosis and treatment. Nevertheless, designing a highly accurate classification model on 31A1/31A2/31A3 fractures from the X-ray is still limited due to the failure of capturing the scale-variant and contextual information. As a result, this paper proposes a deep scale-variant (DSV) network with a hybrid and progressive (HP) loss function to aggregate more influential representations of the fracture regions. More specifically, the DSV network is based on the ResNet and integrated with the designed scale-variant (SV) layer and HP loss, where the SV layer aims to enhance the representation ability to extract the scale-variant features, and HP loss is intended to force the network to condense more contextual clues. Furthermore, to evaluate the effect of the proposed DSV network, we carry out a series of experiments on the real X-ray images for comparison and evaluation, and the experimental results demonstrate that the proposed DSV network could outperform other classification methods on this classification task.

## 1. Introduction

Femur trochanteric fracture has been a common healthcare problem for elderly people, which severely influences the daily life of the injured people. Currently, the most effective way to assist the radiologist in diagnosing this disease is by adopting X-ray or computed tomography (CT) to examine the injured parts and then undergoing reasonable treatments. Especially, in clinical diagnosis, the most commonly used classification criterion for the fracture is the OA/OTA, which divides the fracture into three types: 31/A1, 31/A2, and 31/A3, based on the conditions of the different fractures [1]. In the type of 31/A1, it always comes with pertrochanteric fracture, and in 31/A2, it defines the multifragmentary pertrochanteric fracture, while in 31/A3, it usually represents the reverse obliquity (as shown in Figure 1). Based on this criterion, the orthopaedic surgeon could diagnose the fracture types more precisely and then make the follow-up treatment plan according to different fracture types to achieve the personalized diagnosis. However, in clinical practice, the manual examination for each patient's images is usually a tedious and labor-intensive job. In addition, due to the different clinical experiences of radiologists, the final diagnosis result could be slightly diverse which may be a handicap for the subsequent treatment. Thus, to address those challenges, many attempts of designing the algorithms for the computer-aided system to achieve the automatic classification of the OA/OTA are widely proposed. For example, Aruse et al. [2] designed a three-dimensional computer model which computed the four scaphoid axes to measure the direction and angle of the fracture and then calculated the correlation of different fracture angles to prove that the direction of the fracture inclination was less influential in scaphoid fractures. Basha et al. [3] designed an efficient and automatic bone fracture detection system which combined the enhanced Haar wavelet transform with scale-invariant feature transform (SIFT) to extract the image features and then input them to a neural network for bone fracture classification; the final experimental results indicated that the designed model could gain better classification performance compared with the SIFT method. Yin et al. [4] explored the Tang classification system which was based on the three-dimensional image analysis system to achieve the automatic classification of the femoral intertrochanteric fracture, and it demonstrated that the proposed Tang classification system could be more reliable than other ones in this task. Moreover, in the work [5], it proposed an exemplar pyramid architecture that learned different image features and then classified the fracture types by adopting the classical classifiers. Burns et al. [6] utilized the machine learning approach to create an automated detection and localization computer-aided system by extracting high-level vertebral compression fracture features to gain a high sensitivity classification performance. In [7], the authors extracted the texture and shape features of the vertebral bodies from the median sagittal planes of lumbar spine images and applied different classifiers to classify the osteoporosis or vertebral metastasis fractures. Although those designed methods could effectively improve the efficiency of the diagnosis process and alleviate the workload of the radiologist, the subjective feature definition and selection of those hand-crafted based methods is still a challenging problem.

The article "Deep Scale-Variant Network for Femur Trochanteric Fracture Classification with HP Loss" was retracted in 2023. Reasons: signs of a paper mill; compromised peer review; unreliable results or conclusions.

In recent years, the deep neural network (DNN) has gained promising performance in various computer vision fields and applications [8–14]. Especially, the convolutional neural network (CNN) has been the most prevalent approach in regard to the image classification task. For example, the method in [15] proposed a deep learning architecture that was able to help doctors detect the bone fractures based on the OA/OTA criterion, and the proposed classification model could gain the improvement on average accuracy by 14%. Chung et al. [16] employed a deep learning algorithm to detect and classify proximal humerus fractures on plain anteroposterior shoulder images; it then compared the results with human groups and indicated that the proposed method could obtain superior performance compared with the general physicians and orthopedists. Pranata et al. [17] developed an automatic computer-aided system for fracture detection and classification from the calcaneus CT images; in this system, it extracted the features from coronal, sagittal, and transverse views by adopting CNN, ResNet, and VGG, respectively, and then using the SURF algorithm to classify the bone fracture types. Anami et al. [18] presented a novel architecture to classify diaphyseal tibial fractures by the neural network; it had two main stages, and the first stage aimed to classify the normal and abnormal ones, while the second stage was used to classify the simple, wedge, and complex type of the fracture. Farda et al. [19] used the principle component analysis (PCA) to process the input image and employed the deep neural network to extract the features to gain a better classification performance of calcaneal fracture types. In [20], an artificial intelligence (AI) system was reported to evaluate the performance of classifying knee fractures based on the AO/OTA criterion, and the comparison results demonstrate that the CNN could be utilized for both fracture identification and classification. To achieve the automatic segmentation of fracture regions, the previous work [21] exploited a segmentation model by adopting the Unet structure to segment the wrist fractures, which performed competitive performance at that time. Furthermore, in [22, 23], the authors tried the Inception V3 and Inception-ResNet for efficiently extracting the high-level representations from the fracture regions. After that, Krogue et al. [24] explored the dense network to achieve the placement of the hip fractures and evaluated the performance on the 100-image subset.

In spite of those previous methods having gained promising results on this classification task, those ones are mainly suffering from failing to learn the scale-variant and contextual information from the feature space, which leads to a handicap for achieving a better classification performance. Note that since edge computing device is widely used in healthcare diagnosis or treatment, herein, developing an accurate and timely classification model is essential and valuable to achieve a remote and intelligent diagnosis. To address those above challenges, in this paper, we propose a deep scale-variant network with a hybrid progressive loss function to achieve the automatic classification of the femur trochanteric fracture from X-ray images. Unlike those previous works, our DSV network is based on the ResNet which is widely used in the computer vision field. At the beginning, to capture the scale-variant feature representations, we design a scale-variant (SV) layer, which uses the adaptive convolution layers with the channel attention mechanism to enhance the scale-variant feature learning ability of the network. Furthermore, providing sufficient contextual information or clues of the fracture regions could also be of great importance in the classification of 31A1/31A2/31A3. Thereby, we design a hybrid and progressive (HP) loss for strengthening the influence of the contextual features, which in turn gain a more accurate classification performance. Finally, we conduct a series of exhaustive experiments on the real X-ray images and report the comparison results to effectively validate the effectiveness of the DSV network.

The article "Deep Scale-Variant Network for Femur Trochanteric Fracture Classification with HP Loss" was retracted in 2023. Reasons: signs of a paper mill; compromised peer review; unreliable results or conclusions.

In the following sections, we first introduce the proposed method in Section 2 and then give the descriptions of the experimental data and evaluation metrics in Section 3. Lastly, the comprehensive conclusion is discussed in Section 4.

## 2. Methodology

In this paper, we propose a scale-variant network that could efficiently learn the contextual and scale features from the femur trochanteric region. As illustrated in Figure 2, the whole network is based on the ResNet, which has been widely used in many computer vision fields. Especially, to capture the scale-variant representations, a scaled variant (SV) layer is developed to enhance the feature learning ability of the network. Moreover, a hybrid and progressive (HP) loss function is employed to obtain the highly discriminative deep features from different network levels. In the following sections, we elaborate on the details of SV layer and HP loss.

### 2.1. Network Architecture

Figure 2 shows the overview architecture of the proposed DSV network. Especially, the main backbone of the network is based on ResNet, and we omit the repeated layers for concise display. Compared with the ResNet, the DSV network mainly contains two different parts. Specifically, the first part is the SV layer, which extracts the deep scale-variant features consecutively. The second part is the HP loss, which is calculated to emphasize the contextual and discriminative regions. With the help of those two parts, inputting an X-ray image of the femur trochanteric, it first generates the coarse feature map through each residual feature learning part and then delivers the generated one to SV layer for obtaining the scale-variant representations. Note that considering the complexities of the network, we only deploy SV layer before each residual learning phase. Finally, the extracted high-level features enter into a fully connected (FC) layer with the cross-entropy loss to impel the network focus on the universal parts. The proposed HP loss calculates the diversities from different network levels to highlight the discriminative contextual regions.

The article "Deep Scale-Variant Network for Femur Trochanteric Fracture Classification with HP Loss" was retracted in 2023. Reasons: signs of a paper mill; compromised peer review; unreliable results or conclusions.

### 2.2. Scale-Variant Layer

Although the hierarchical layers of the network enable it to extract the deep features, it is still limited by the fixed filter size, which leads to incorrect classification of the fracture regions. To address this challenge, in our DSV network, we develop an SV layer, which deploys it before each residual learning phase to adaptively and progressively extract the scale-variant representations. The detailed structure of the SV layer is shown in Figure 3; it obeys the residual connection to facilitate the training process. Specifically, we denote the input feature from the previous residual learning phase as *𝔽* ∈ *ℝ*^*H*×*W*×*C*^ where *H*, *W*, *C* denote the height, width, and channel numbers of *𝔽*, respectively. Then, in the SV layer, it first passes *𝔽* into three separate 1 × 1 layers to compress the feature maps, which denotes the output feature map as *𝔽*_1_ ∈ *ℝ*^*H*×*W*×*c*/2^, *𝔽*_2_ ∈ *ℝ*^*H*×*W*×*c*/2^, and *𝔽*_3_ ∈ *ℝ*^*H*×*W*×*c*/2^, respectively. Subsequently, *𝔽*_1_ is directly delivered into the channel attention (CA) module, which aims to further prune the feature map from the channel level. Mathematically, split *𝔽*_1_ into channel level expression, which can be denoted as

(1) $$\begin{array}{c} F_{1}=\left[F_{1}\left(1\right),F_{1}\left(2\right),\ldots ,F_{1}\left(c\right),\ldots ,F_{1}\left(C/2\right)\right], \end{array}$$

where *𝔽*_1_(*c*) indicates the *c*-th channel feature map of *𝔽*, *c* ∈ {1,2,…, *C*/2}. Then, the *𝔽*_1_(*c*) is first applied by a global average pooling over the full channel feature map, and the operation of GAP could be given as

(2) $$\begin{array}{c} t_{c}=\frac{1}{H\times W}\overset{H}{\sum }\overset{W}{\sum }F_{c}, \end{array}$$

where the parameter of *t*_*c*_ represents the overall factor value of *c*-th feature map channel. Then, a gating mechanism is utilized to learn the dependencies of each feature channel, which can be formulated as

(3) $$\begin{array}{c} t^{\prime }=\sigma \left(W\delta \left(W^{\prime }t\right)\right), \end{array}$$

where *t*′ indicates the importance factor, *𝕎* and *𝕎*′ are the weights of two fully connected layers, separately, and *δ*(*·*) represents the ReLU activation which could be given as

(4) $$\begin{array}{c} \delta \left(x\right)=\max\left(0,x\right), \end{array}$$

where *σ*(*·*) denotes the sigmoid activation function, and it can be defined as

(5) $$\begin{array}{c} \sigma \left(x\right)=\frac{1}{1+e^{-x}}. \end{array}$$

After that, the gained importance factor *t*_*c*_′ multiplies with *𝔽* to obtain the enhanced feature map *𝔽*′:

(6) $$\begin{array}{c} F_{1}^{\prime }=F_{1}\cdot t^{\prime }. \end{array}$$

Notably, in order to learn the scale-variant features more efficiently, before applying the CA to *𝔽*_2_ and *𝔽*_3_, we deliver *𝔽*_2_ to a 3 × 3 convolution layer and feed *𝔽*_3_ through two 3 × 3 convolution layers, respectively. Afterwards, denote the outputs of CA module of *𝔽*_2_ and *𝔽*_3_ as *𝔽*_2_′ and *𝔽*_3_′, and then those three scale-variant representations (*𝔽*_1_′, *𝔽*_2_′, *𝔽*_3_′) are fused as follows:

(7) $$\begin{array}{c} F_{sv}=\tau \left\{F_{1}^{\prime },F_{2}^{\prime },F_{3}^{\prime }\right\}, \end{array}$$

where *τ*(*·*) represents the concatenation operation. By adopting the SV layer, the network is more effective to extract the scale-variant features, which is able to further improve the classification performance of the DSV network. Moreover, to further explore the contextual information of the image, we employ a hybrid and progressive loss, which could efficiently enhance the network to spotlight the discriminative femur trochanteric fracture regions.

The article "Deep Scale-Variant Network for Femur Trochanteric Fracture Classification with HP Loss" was retracted in 2023. Reasons: signs of a paper mill; compromised peer review; unreliable results or conclusions.

### 2.3. Hybrid and Progressive Loss

To efficiently extract more contextual information from the femur trochanteric fracture regions, we develop a hybrid and progressive loss function *L*_*HP*_:

(8) $$\begin{array}{c} {ℒ}_{HP}={ℒ}_{ce}+\mu \times {ℒ}_{sp}, \end{array}$$

where *L*_*ce*_ denotes the cross-entropy loss function, *L*_*sp*_ is the side progressive loss function, and *μ* is a weighting hyperparameter to balance those two loss functions. More specifically, *L*_*ce*_ could be defined as

(9) $$\begin{array}{c} {ℒ}_{\text{ce }}=\sum_{k=1}^{N}y_{k}\log\;p_{k}+\sum_{j=k}^{N}\left(1-y_{k}\right)\log\left(1-p_{k}\right), \end{array}$$

where *p*_*k*_ is the predicted probability for class *k*, *y*_*k*_ is the true label, and the value of *N* is 3. Note that the value of *p*_*k*_ is calculated from the FC layer with the softmax activation function:

(10) $$\begin{array}{c} \psi {\left(s\right)}_{i}=\frac{e^{s_{i}}}{\sum_{n=1}^{3}e^{s_{n}}}, \end{array}$$

where *s*_*i*_ is the output feature map from the FC layer. Furthermore, *L*_*sp*_ is a combined one which is formulated as

(11) $$\begin{array}{c} {ℒ}_{sp}=\sum_{m=1}^{M}{ℒ}_{p}, \end{array}$$

where the value of *M* is set as 3; considering the trade-off between network complexity and efficiency, ℒ_*p*_ is gained by

(12) $$\begin{array}{c} {ℒ}_{p}=\rho \left(\gamma \left({ℱ}_{m}\right)\right), \end{array}$$

where *γ*(*·*) is the cross channel max-pooling [25] to merge the feature map to the dimension of *H* × *W* × 3, *ρ* is the global average pooling, and ℱ_*m*_ is the feature map from last *m*-th residual block of the network. By aggregating the contextual clues with a progressive learning mode, it forces the network to produce more abstract and essential information, thus leading to a better classification performance.

The article "Deep Scale-Variant Network for Femur Trochanteric Fracture Classification with HP Loss" was retracted in 2023. Reasons: signs of a paper mill; compromised peer review; unreliable results or conclusions.

## 3. Experiment

To demonstrate the effectiveness of the proposed model, in this section, we validate our proposed model with real femur trochanteric fracture images. Besides, we carry out a series of experiments to explore the influence of different configurations on classification performance. Extensive experimental results demonstrate that the proposed DSV network could gain competitive classification performance compared with other state-of-the-art approaches. In the following content, we will provide detailed descriptions of the experimental dataset, implementation details, evaluation metrics, and experimental results.

### 3.1. Dataset

For the evaluation dataset, we adopt three types of data (31/A1, 31/A2, and 31/A3), with the amount of 117, 125, and 128, separately. Especially, the max/min age of the evaluated dataset is 91 and 26, respectively, and the mean age of the dataset is 65. For accurate evaluation of the proposed model, the types of the experimental dataset are confirmed by three orthopaedic specialists with experience over 5 years based on the AO/OTA criterion. Notably, the input image is resized to 512 × 512 and the region of interest (ROI) of the original image is cropped for reducing the computational complexity.

### 3.2. Implementation Details

In our validation experiments, we implemented the network by the PyTorch platform with the NVIDIA GTX2070 graphics processing unit (GPU). For the network training, we use the Adam optimizer and set the initial learning rate as 0.001 in the first 60 epochs and then decay the value by 0.01 for the following 30 epochs. To increase the amount of the data, we use data augmentation such as random flipping, rotation, cropping, and padding to generate more training data. Particularly, the batch size of our model is 5, and before inputting the ROI image to the network, we resize them to 512 × 512.

The article "Deep Scale-Variant Network for Femur Trochanteric Fracture Classification with HP Loss" was retracted in 2023. Reasons: signs of a paper mill; compromised peer review; unreliable results or conclusions.

### 3.3. Evaluation Metrics

In this section, we evaluate our model by employing accuracy, sensitivity, specificity, and the area under the curve (AUC) score. The accuracy is the measurement of the true predicted values, which can be formulated as

(13) $$\begin{array}{c} \text{accuracy}=\frac{TP+TN}{TP+FP+TN+FN}, \end{array}$$

where TP, TN, FP, and FN represent the true positive, false positive, true negative, and false negative, respectively. The sensitivity denotes the ability to identify the true positives, and it can be defined as

(14) $$\begin{array}{c} \text{sensitivity}=\frac{TP}{TP+FN}, \end{array}$$

while the specificity indicates the ability to identify the true negatives, which could be given as

(15) $$\begin{array}{c} \text{specificity}=\frac{TN}{TN+FP}. \end{array}$$

Specifically, the AUC score is the classical metric to evaluate the performance of the classifier; the higher the score of the AUC is, the better performance the model would gain.

### 3.4. Impact of Different Data Samples

Table 1 reports the comparison results on different data samples, where it is divided into 20%, 40%, 60%, 80%, and 100% of the total data samples. Note that we do not test smaller percent (<20%) of the data samples, since it could be hard for the network to be convergent. From the comparison results, we can observe that the best performance is achieved by adopting 100% of data samples, which could be explained that more data samples could provide more robust representations that further boost the classification performance. Moreover, with the increasing number of data samples, the classification performance is stably improving which is also consistent with the prementioned hypothesis.

### 3.5. Ablation Study of Different Components

In this section, we employ extensive experiments to conduct the ablation study of different components. As illustrated in Table 2, we explore three comparisons which are “ResNet,” “ResNet + SV,” “ResNet + HP,” “ResNet + SV + HP,” respectively. Here, “+ SV,” “+ HP,” and “+ SV + HP” denote the network with the scale-variant layer, hybrid and progressive loss, and simultaneous two parts. From the results, we observe that the best performance is obtained by “ResNet + SV + HP” with a score of 90.2%, 88.9%, 86.5%, and 0.98 on the accuracy, sensitivity, specificity, and AUC, respectively. Moreover, compared with different network settings, “ResNet + SV” could achieve better performance than “ResNet + HP,” which indicates that the scale-variant features could have more significant impact compared with the contextual clues on this classification task.

### 3.6. The Influence of Different Branch Numbers of SV Layer

In our SV layer, we utilize three branches to capture the scale-variant features; however, it could be flexible to select the numbers of the branches. Therefore, in this section, we carry out experiments to evaluate the influence of different branches of the SV layer. The comparison result is shown in Table 3, and there are four branch numbers (1, 2, 3, 4) for comparison. At the beginning, it is obvious that using more branches could improve the classification performance; however, when the number of the branch is bigger than 3, the performance is not efficiently improved on those four metrics. Therefore, to balance the trade-off between the complexity and performance, we still adopt the 3 branches as the final set of SV layer. In summary, the final performance of applying 3 branches is 90.2%, 88.9%, 86.5%, and 0.98 on the accuracy, sensitivity, specificity, and AUC, separately.

The article "Deep Scale-Variant Network for Femur Trochanteric Fracture Classification with HP Loss" was retracted in 2023. Reasons: signs of a paper mill; compromised peer review; unreliable results or conclusions.

### 3.7. The Performance of Various HP Loss Settings

In order to further evaluate the influence of HP loss, especially the calculated location on the network, in this section, we conduct a series of experiments to validate its effect. Since we only calculate the outputs of the last three residual blocks of the DSV network, here we denote “HP-1,” “HP-2,” and “HP-3” as the third to last, next to last, and last of the residual block, while “HP-o” and “HP-123” represent the DSV network without or with the HP loss. As illustrated in Table 4, the comparison result demonstrates that using the HP loss with any location of the DSV network could boost its classification performance compared with “HP-o,” and furthermore, it is obvious that the best performance is achieved by “HP-123.”

### 3.8. Comparison with Other Methods

In this section, we compare our proposed DSV network with other classification methods to evaluate its effectiveness.  Table 5 lists the comparison results, and here we employ some baseline methods such as Inception V4 [26], ResNet [27], DenseNet [28], SKNet [29], Res2Net [30], and DDA [31]. It is evident that compared with other classification methods, our DSV network gains more accurate classification on the four evaluation metrics. It could be explained that with the designed SV layer and HP loss, the DSV network has more powerful feature ability on the scale-variant and contextual clues, which leads to better classification performance.

## 4. Conclusion

In this paper, we have proposed a DSV network for the automatic classification of the femur trochanteric fracture. The DSV network aggregates the scale-variant representation through the SV layer and learns the contextual clues by the HP loss from different depths of layers. To evaluate the effectiveness of the DSV network, we perform extensive experiments on the real femur trochanteric fracture of X-ray images, and the exhaustive comparison results demonstrate that the proposed DSV network could be superior to other recent image classification methods with higher classification performance. In the future work, we will mainly focus on employing our model on different modalities images such as magnetic resonance imaging (MRI) and computed tomography (CT) to explore the effectiveness of the proposed model. Moreover, we would try to deploy our model with lighter one on the edge computing device to help achieve the remote diagnosis efficiently.

The article "Deep Scale-Variant Network for Femur Trochanteric Fracture Classification with HP Loss" was retracted in 2023. Reasons: signs of a paper mill; compromised peer review; unreliable results or conclusions.

## Figures and Tables

**Figure 1:** The data samples of 31/A1, 31/A2, and 31/A3.

**Figure 2:** The main architecture of the DSV network: *L*_*p*_ is one part of the HP loss, and CCMP and GAP denote the cross channel max-pooling layer and global average-pooling layer, respectively.

**Figure 3:** The structure of the SA layer.

**Table 1:** The impact of different data samples.

Data samples (%)	Accuracy (%)	Sensitivity (%)	Specificity (%)	AUC
20	85.2	85.1	82.0	0.83
40	85.6	86.1	83.1	0.85
60	86.7	86.9	83.6	0.88
80	88.8	87.3	85.3	0.94
100	90.2	88.9	86.5	0.98

**Table 2:** The comparison results of different components of DSV network.

Components	Accuracy (%)	Sensitivity (%)	Specificity (%)	AUC
ResNet	87.5	86.7	81.9	0.87
ResNet + SV	89.3	87.5	85.6	0.95
ResNet + HP	88.9	87.3	85.4	0.94
ResNet + SV + HP	90.2	88.9	86.5	0.98

**Table 3:** The comparison results of different branch numbers of SV layer.

Branch numbers (BNs)	Accuracy (%)	Sensitivity (%)	Specificity (%)	AUC
ResNet	87.5	86.7	81.9	0.87
BNs = 1	88.7	87.5	85.3	0.94
BNs = 2	88.9	88.2	85.5	0.96
BNs = 3	90.2	88.9	86.5	0.98
BNs = 4	90.2	88.6	86.4	0.97

**Table 4:** The performance of various HP loss settings.

	Accuracy (%)	Sensitivity (%)	Specificity (%)	AUC
HP-o	89.3	87.5	85.6	0.95
HP-1	89.3	87.8	85.3	0.95
HP-2	89.7	88.2	85.7	0.96
HP-3	89.8	88.7	85.8	0.97
HP-123	90.2	88.9	86.5	0.98

**Table 5:** The comparison results with other methods.

Method	Accuracy (%)	Sensitivity (%)	Specificity (%)	AUC
Inception V4 [26]	87.8	86.1	82.3	0.86
ResNet [27]	87.5	86.7	81.9	0.87
DenseNet [28]	87.2	86.3	83.4	0.91
SKNet [29]	87.1	86.8	83.6	0.92
Res2Net [30]	88.2	87.7	85.7	0.95
DDA [31]	88.9	87.6	85.9	0.97
DSV	90.2	88.9	86.5	0.98
